The article "Diagnostic Significance of 18F-FDG PET/CT Imaging Coupled with Magnetic Resonance Imaging of the Entire Body for Bone Metastases" was published in 2022. Journal: Contrast Media Mol Imaging.

# Diagnostic Significance of 18F-FDG PET/CT Imaging Coupled with Magnetic Resonance Imaging of the Entire Body for Bone Metastases

**DOI:** 10.1155/2022/7717398

**Published:** 2022-09-27

**Authors:** Huimin Guo, Zhiwen Zhang, Li Wang, Shuzhan Yao, Shuaishuai Xu, Shulin Ma, Songtao Liu

**Affiliations:** ^1^Department of Nuclear Medicine, Shandong Provincial Hospital Affiliated to Shandong First Medical University, Jinan 250021, China; ^2^Department of Ultrasound, Shandong Provincial Hospital Affiliated to Shandong First Medical University, Jinan 250021, China; ^3^Department of Rehabilitation, Shandong Provincial Hospital Affiliated to Shandong First Medical University, Jinan 250021, China

## Abstract

**Objective:**

To see if 18F-fluorodeoxyglucose positron emission tomography/computed tomography (18F-FDG PET/CT) imaging paired with MR diffusion imaging can help doctors diagnose bone metastases.

**Methods:**

From September 2020 to December 2021, a total of 30 individuals with probable bone metastases were recruited for the trial. With an average interval of four days, MAGNETIC resonance whole-body diffusion imaging (MR whole-body diffusion imaging) was performed on each of the 30 patients who had 18F-FDG PET/CT. The SUVmax values of the group with bone metastases were compared to those of the group without bone metastases. In this study, 18F-FDG PET/CT imaging, MR whole-body diffusion imaging, and their combination were examined. The researchers compared the results when 18F-FDG PET/CT imaging, whole-body MRI diffusion scans, and their combination indicated abnormal bone lesions. By comparing the diagnostic efficacy of 18F-FDG PET/CT imaging, MR whole-body diffusion imaging, and their combination, as well as accuracy, sensitivity, and specificity, the three techniques for diagnosing bone metastases will be evaluated for diagnostic usefulness. Results: the SUV max values of patients with bone metastases were significantly different from those of patients without bone metastases, as determined by 18F-FDG PET/CT imaging (*P* < 0.05). Using 18F-FDG PET/CT imaging, MR whole-body diffusion imaging, and their combined detection of aberrant bone lesions in various areas, we found statistically significant differences.

**Conclusion:**

The use of 18F-FDG PET/CT imaging in conjunction with MR whole-body diffusion imaging in the diagnosis of bone metastases can be very helpful.

## 1. Background

Malignant tumors can spread from another part of the body to the bone in a variety of ways, where they can then grow and develop into new cancers called bone metastases [1], which are particularly common in breast, prostate, lung, and thyroid cancers. According to statistics, about 3/4 of cancer patients die of bone metastasis [2]. If the location and symptoms of the tumor are not obvious to the patient, metastatic bone tumors are easily misdiagnosed and even diagnosed and treated as primary bone tumors [3]. MAGNETIC resonance whole-body diffusion imaging (MR whole-body diffusion imaging) makes use of the characteristic of limited movement of water molecules in tumor tissue cells so that bone metastases show high signal on DWI and are diagnosed [4]. This highly advanced technology plays a vital role in the diagnosis and staging of cancer tumors. 18 f-fluoro deoxidization glucose/electron-positron emission computed tomography (CT) imaging computed tomography (18f-fluorodeoxyglucose positron emission tomography/computed tomography, 18F-FDG PET/CT matched the anatomical information provided by CT with functional PET images, and a single examination can fully show the distribution, size, number, and metabolic activity of MM systemic bone lesions and extraosseous lesions. 18F-FDG PET/CT can identify the degree of glucose absorption by the tumor and indirectly reflect the activity of the lesion [5]. The application of 18F-FDG PET/CT imaging and whole-body diffusion imaging in the diagnosis of bone metastases is still under investigation to evaluate the diagnostic value of 18F-FDG PET/CT and whole-body magnetic resonance diffusion imaging and their combination in bone metastases. Thus, the findings are as follows.

The article "Diagnostic Significance of 18F-FDG PET/CT Imaging Coupled with Magnetic Resonance Imaging of the Entire Body for Bone Metastases" was published in 2022. Journal: Contrast Media Mol Imaging.

## 2. General Information and Methods

### 2.1. General Information

From September 2020 to December 2021, 30 individuals with probable bone metastases were recruited for the trial. With a mean age of 53.17 ± 2.65 years, according to the survey, there were 19 men and 11 women between the ages of 48 and 61. All 30 patients had 18F-FDG PET/CT and MR whole-body diffusion imaging at intervals averaging four days. Each participant was given a signed informed consent form. In conformity with the principles described in the Declaration of Helsinki, the research was conducted. Hospital's Medical Ethics Committee has given its support to this research.

### 2.2. Included and Excluded Criteria

Inclusion criteria are as follows: (1) age: >18, (2) life expectancy >12 months, (3) suspected bone metastases were diagnosed by imaging, (4) no contraindications of examination, (5) good compliance, and (6) clinical data are complete, and relevant imaging and laboratory tests are true and accurate.

Exclusion criteria are as follows: (1) prior to admission, there was a history of chemotherapy, radiotherapy, surgery, and other related treatments, (2) accompanied by severe liver and kidney dysfunction, (3) tumors at other sites and distant metastasis, (4) the presence of serious organic diseases, and (5) history of severe acute infection during admission.

The article "Diagnostic Significance of 18F-FDG PET/CT Imaging Coupled with Magnetic Resonance Imaging of the Entire Body for Bone Metastases" was published in 2022. Journal: Contrast Media Mol Imaging.

### 2.3. Methods

18F-FDG PET/CT imaging: 64-row PET/CT (Siemens Healthcare, Erlangen, Germany, Biograph mCT). Radiopharmaceutical 18F-FDG, i.e., fluoro-deoxyglucose radiopharmaceutical purity >95%. Before the assessment, the patient had been fasting for six to eight hours, and his blood glucose was within 7.0 mmol/L. It was injected into the cubital vein following a 10-minute supine rest period. It took 60 minutes of recumbent rest before the entire body 18F-FDG PET/CT examination could begin. Before scanning, the patient's bladder was drained. The CT positioning scan was carried out first, and the parameters were set as tube voltage: 120 KV, tube current: reference mAs, pitch: 0.8, reconstruction layer thickness: 3.0 mm, and interval: 2.0 mm. Then, PET images of corresponding parts in line were collected with an ultrahigh energy collimator, and the parameters were set as energy peak: 511 keV, layer thickness: 3.0 mm, window width: 20%, and collection time: 2 min/bed. Scanning of the entire body was carried out on a regular basis, and limbs were additionally scanned if necessary due to pathological conditions. After attenuation correction and iterative reconstruction of the PET image from the original image data, a 3d image was automatically generated on the workstation, and the sectional, sagittal, and coronal plane fault maps were obtained. Moreover, image fusion with the same machine positioning CT image was obtained.

Magnetic resonance body diffusion imaging: magnetic resonance imaging technology can obtain the physical characteristics and microstructure of biological tissues by detecting the diffusion characteristics of water molecules so as to provide biological and clinical medical information. It has the advantages of noninvasiveness, and there is no need to use an exogenous contrast agent. Recent advances in magnetic resonance technology show that diffusion imaging research is one of the most important and clinically relevant fields. A Signa ExciteTM magnetic resonance imaging machine (GE medical systems) emits and receives signals from a body coil. Immobilization and a quiet breathing pattern were maintained for the patient. Foot first, 8 sections of imaging were performed from the head to the middle leg, 26 layers were collected in each section, and the imaging distance was 1664 mm in total. After removing the overlap between segments, an effective imaging distance of 1417 mm remains. The parameters were set at time of echo (TE): 62.5 ms, time of repetition (TR): 6000 ms, time of inversion (TI): 220 ms, number of excitation (NEX): 3 times, field of view (FOV): 38 cm × 38 cm, matrix: 96×96, B value: 800 mm2/s, layer thickness: 8 mm, and no interval imaging. The acquisition time of each segment is 150s, and the total acquisition time is about 30 min. All axial plane images were spliced using the connection technology, and then the maximum signal projection image was obtained by 3D reconstruction, and the final diagnostic image was obtained by black and white inversion.

The article "Diagnostic Significance of 18F-FDG PET/CT Imaging Coupled with Magnetic Resonance Imaging of the Entire Body for Bone Metastases" was published in 2022. Journal: Contrast Media Mol Imaging.

### 2.4. Diagnostic Criteria for Bone Metastases

Patients were split into two categories based on the gold standard for diagnosing bone metastases: those with and those without bone metastases.

Negative must meet more than one of the following conditions:

1. The abnormal radioactive distribution of the lesions was showed during the time when initial imaging disappeared, and the patient had no symptoms such as bone pain from beginning to end
2. CT showed no osteolytic or osteogenic changes
3. MRI showed no abnormal signal

Positive must meet more than one of the following conditions:

1. Abnormal bone lesions were confirmed as bone metastases by puncture or surgical pathology;
2. The gold standard for relative lesions in metastatic cancers was abnormal 18F-FDG PET/CT imaging or positive results on conventional MR T1WI and fat compression T2WI. Combining the results of ordinary film X-rays, CT scans, MRIs, and radionuclide bone imaging allowed for a comprehensive diagnosis.
3. For abnormal bone lesions without histological or pathological findings, the above imaging examinations are still difficult to determine, and the response to radiotherapy and chemotherapy or follow-up for more than 3 months can be used to confirm the diagnosis.

### 2.5. Image Analysis

Imaging scans were examined separately by two experts in the field of radiology using only 18F-FDG PET/CT and MR whole-body diffusion imaging scans.18F-FDG PET/CT imaging: higher uptake of surrounding normal soft tissue, SUVmax>2.5, nodules, clumps or strips, diffuse or focal, and ≥2 bone scan concentration indicated the presence of abnormal bone foci. MR whole-body diffusion imaging: the uneven size and nodular hyperintensity of the skeletal system in the image were recorded as bone abnormalities. The skeletal system within the imaging range was divided into 8 regions, and the location and number of abnormal bone foci in the images obtained by two imaging methods in each region were recorded. Finally, the above physicians combined the two imaging methods to interpret the images and determine the number of suspected bone metastases. Sensitivity = true positive/(true positive + false negative)×100%; specificity = true negative/(true negative + false positive)×100%.

The article "Diagnostic Significance of 18F-FDG PET/CT Imaging Coupled with Magnetic Resonance Imaging of the Entire Body for Bone Metastases" was published in 2022. Journal: Contrast Media Mol Imaging.

### 2.6. Observation Indicators

1. When comparing groups with and without bone metastases, the SUVmax values were dramatically different.
2. Comparing bone lesions in different sections of the body may be performed with 18F-FDG PET/CT and MR whole-body diffusion imaging.
3. All parts of the body, including skull, clavicle and sternum, shoulder blade, ribs, spine, pelvis, femoral, tibiofibular, the presence of moth-eaten, granular, punctured –bone-soluble lesions are regarded as Imaging aberrant bone lesions.
4. The diagnostic usefulness of 18F-FDG PET/CT imaging can be evaluated. The diagnostic efficacy of the three methods was compared, including sensitivity and specificity.

### 2.7. Statistical Analysis

Statistical analysis was carried out with the help of SPSS 22.0. There was a statistical comparison between the data groups using *n* (percentage) and a *χ*2 test to describe the statistical data. It was decided to use the consistency test and the area under the ROC curve. AUC in bone metastases was used to evaluate the diagnostic impact of 18F-FDG PET/CT imaging, MR whole-body diffusion imaging, and their combination. The difference was statistically significant when *P* < 0.05.

## 3. Results

### 3.1. Bone Metastasis Group and Nonbone Metastatic Group SUVmax Values

Using 18F-FDG PET/CT imaging, the SUV max value was significantly greater (*P* < 0.05) in the bone metastatic group than in the nonbone metastasis group (Figure 1).

BM: bone metastasis group and N-BM: nonbone metastasis group.

### 3.2. 18F-FDG PET/CT Imaging, MR Whole-Body Diffusion Imaging and Their Combined Examination of Abnormal Bone Lesions in Different Parts of the Body

In 25 individuals, a total of 115 worrisome bone metastases were found using both approaches. 18F-FDG PET/CT imaging detected 87 worrisome bone metastases, and MR whole-body diffusion imaging detected 85 suspicious bone metastases. A total of 95 places suspicious bone metastases were found by combining the two methods. A statistically significant (*P* < 0.05) difference in the number of suspicious bone metastases observed in Table 1 of the *χ*2 test findings was found between 18F-FDG PET/CT, MR whole-body diffusion imaging, and their combined detection of bone metastases (Figure 2).

### 3.3. 18F-FDG PET/CT, MR Whole-Body Diffusion Imaging, and Their Combination

There were 26 and 87 benign and malignant tumors correctly diagnosed using 18F-FDG PET/CT imaging and MR whole-body diffusion imaging, respectively, which were consistent with the gold standard results (Figure 3), respectively, 29, 85, 36, and 95, as shown in Table 2.

### 3.4. Analysis of the Diagnostic Usefulness of 18F-FDG PET/CT Imaging, MR Whole-Body Diffusion Imaging, and Their Combination

The combined sensitivity (97.93%), specificity (92.31%), and AUC (0.856) were significantly higher than those of 18F-FDG PET/CT imaging (89.69%, 66.67%, and 0.747) and MR whole-body diffusion imaging (87.63%, 74.36%, and 0.724), and the difference was statistically significant, as shown in Table 3 and Figure 4.

The article "Diagnostic Significance of 18F-FDG PET/CT Imaging Coupled with Magnetic Resonance Imaging of the Entire Body for Bone Metastases" was published in 2022. Journal: Contrast Media Mol Imaging.

## 4. Discussion

It has been reported that most patients have bone metastasis during or after treatment, and different symptoms may occur according to different sites of metastasis; the most common site of metastasis is bone [6]. Its signs are systemic consumption symptoms, local pain of metastasis, compression symptoms, pathological fracture, and so on. For example, local masses are the first to be found in tumors that metastasized to limb bones, and when metastatic bone cancers spread to the trunk, pain is the most common symptom [7]. In certain cases, patients with a primary malignant tumor exhibited symptoms of metastasis during or after therapy, even if they had no prior history of the condition. It is difficult to diagnose cancer in patients who have no history or indications of the initial tumor, and the first symptom is usually metastasis [8]. Patients' quality of life can be improved by preventing or delaying bone-related occurrences, such as bone metastases. Bone metastases can only be diagnosed by using signs with high sensitivity and specificity. The earlier bone metastases are discovered and treated, the better the chances for a patient's life are for them to be prevented or delayed.

At present, there are many general imaging methods to diagnose bone metastases. X-ray examination is a common means of imaging examination, and the scope and shape of lesions can be seen more intuitively in the four limb bones with less overlap. Bone metastases with overlapping tissues might, however, be difficult to identify. CT is a routine item for local bone examination. It is a tomography, which can effectively avoid structural overlap and has high density and spatial resolution. It is difficult and unreliable to detect early bone metastasis with microbone metastases because of these limitations [9, 10]. PET/CT imaging using 18F-FDG combines functional and anatomical images to locate a lesion's specific location and highlight microscopic characteristics such as the bone cortex and trabecula in the surrounding tissue. At the same time, glucose uptake in bone metastasis can be displayed, and whole-body imaging can be used to understand the extent of bone metastasis, the metabolic activity of tumor tissue, and other organ metastases at a time [11]. MR whole-body diffusion imaging (MRIS) indirectly reflects the changes in tissue microstructure by scanning the limited information of diffusion movement of water molecules in cells in vivo. Therefore, MR whole-body diffusion imaging can not only show the lesions of bone metastases but also reflect the involvement of bone marrow tissues and cells [12].

The article "Diagnostic Significance of 18F-FDG PET/CT Imaging Coupled with Magnetic Resonance Imaging of the Entire Body for Bone Metastases" was published in 2022. Journal: Contrast Media Mol Imaging.

The integration of functional and anatomical images is possible with the use of 18F-FDG PET/CT. These alterations in form and density, as well as their metabolic state, can be used to generate a differential diagnosis of the sick vertebral body [13]. SUVmax values of bone metastasis and nonbone metastasis groups were statistically significant using 18F-FDG PET/CT imaging. The noninvasive measurement of tumor effectiveness may be enhanced by the use of SUVmax. An 18F-FDG PET/CT scan can measure tumor metabolic activity by determining the tumor cells' glucose metabolism level. 18F-FDG is a glucose analog, which can reflect glucose utilization in living tissues, and is the most commonly used imaging agent in clinics. Its imaging mechanism is that after intravenous injection, 18F-FDG is deposited by ion exchange, chemisorption, or combination with organic matrix, and local aggregates of different sizes are carried out according to the active level of bone salt metabolism and blood flow [14]. Studies have found that the site of bone metastasis has abundant blood flow and vigorous metabolism, resulting in more local concentration and presenting as an abnormal concentration area [15]. It has been reported that tumor bone metastasis mostly develops outward from the inside of the bone marrow, first invading the bone marrow and then the bone cortex [1 6]. For the purpose of detecting abnormal bone lesions, this study compared MR whole-body diffusion imaging with 18F-FDG PET/CT imaging and found statistically significant differences. Analysis shows that the range of MR whole-body diffusion imaging is limited. However, obvious and suspicious bone metastases could be found in areas with high bone marrow content, high cellular water content, and slow and abundant blood transport. PET/CT has the advantages of high probe detection efficiency, strong spatial resolution of the image, short acquisition time, and good reliability of quantitative analysis. The imaging of suspicious bone metastases can be found in areas with less bone marrow content and prone to early destruction of the bone cortex, and the simultaneous use of both can make up for their disadvantages [17, 18]. Metabolic features of tumor metastases are often identical to those of the parent tumor [19]. 18F-FDG PET/CT, MR whole-body diffusion, and their combined diagnosis of benign and malignant lesions were statistically significant, and AUC values were considerably higher than 18F-FDG PET/CT and MR whole-body diffusion alone. Noninvasive imaging includes MRI whole-body diffusion and 18F-FDG PET/CT. They have distinct advantages when it comes to determining the extent to which cancers have invaded various organs and tissues throughout the body. While lytic bone destruction was the most common source of false negatives, the study found that other factors such as osteoarthritis, previous fractures, and surgery were more common causes of false positives, which were the actual reflection of limitations. Inflammatory cells assimilate 18F-FDG less than malignant tumors. Studies have shown that nodular or lumpy concentration along the fracture line with diffuse mild concentration of the sacrum is the uptake characteristic of PET/CT [20]. Malignant tumors can stimulate the release of a variety of cytokines, inhibit osteoclasts, and activate osteoblasts, leading to excessive osteogenesis and abnormal bone structure on imaging [21]. This analysis suggests that highly invasive tumors can lead to local bone tissue blood flow interruption or reduced bone salt metabolism, thus presenting defects. However, due to the limitation of spatial resolution and the influence of chest respiratory motion artifacts and partial volume effect, the smaller lesions cannot be displayed, and the image is susceptible to the interference of artifacts, leading to a decrease in diagnostic accuracy [22, 23].

18F-FDG PET/CT imaging with MR whole-body diffusion imaging is superior to any single technique for diagnosing bone metastases. Bone metastases can be diagnosed and evaluated more effectively if these two approaches are used together. Due to a small number of instances, the lack of big sample data, and the lack of multicenter research data, it is difficult to draw conclusions, and it is difficult to conduct a more detailed statistical analysis on the imaging characteristics of various pathological types of bone metastasis, which needs to be verified by the further study of case data.

The article "Diagnostic Significance of 18F-FDG PET/CT Imaging Coupled with Magnetic Resonance Imaging of the Entire Body for Bone Metastases" was published in 2022. Journal: Contrast Media Mol Imaging.

## Figures and Tables

**Figure 1:** SUV max values of two groups.

**Figure 2:** Abnormal bone lesions in different parts of the body.

**Figure 3:** Gold standard for diagnosing bone metastases with different imaging methods.

**Figure 4:** Diagnostic effect of imaging methods.

**Table 1:** Comparison of 18F-FDG PET/CT imaging, MR whole-body diffusion imaging, and their combined examination of abnormal bone lesions in different parts of the body.

Parts of the body		18F–F DG PET/CT imaging		Magnetic resonance whole-body diffusion imaging		Two combined	
		+	-	+	-	+	-
Skull	5	2	0	2	0	2	0
Clavicle and sternum	4	2	0	2	2	2	0
Shoulder blade	5	3	1	4	0	4	0
Ribs	38	27	4	26	3	30	1
Spine	49	32	5	33	3	35	1
Pelvis.	19	12	1	10	2	13	1
Femoral	12	6	1	5	0	6	0
Tibiofibula	4	3	1	3	0	3	0
Total	136	87	13	85	10	95	3

+: true positive; -: false positive.

**Table 2:** Comparison of 18F-FDG PET/CT imaging, MR whole-body diffusion imaging, and their combined diagnosis with the “gold standard” diagnosis of bone metastases.

Gold standard	PET/CT imaging		MR imaging		Two combined		Total
	+	-	+	-	+	-	
+	80	10	81	2	93	0	90
-	7	3	4	8	2	3	7

**Table 3:** MR whole-body diffusion imaging and their combined examination techniques were examined to determine the diagnostic usefulness of 18F-FDG PET/CT images.

Diagnosis way	AUC (95%CI)	Cut-off value	Sensitivity	Specificity
18 F - FDG PET/CT imaging	0.747 (0.613–0.857)	0.734	(87/97), 89.69%	(26/39), 66.67%
Magnetic resonance whole-body diffusion imaging	0.724 (0.577–0.832)	0.704	(85/97), 87.63%	(29/39) 74.36%
Two combined	0.856 (0.691–0.943)	0.890	(95/97), 97.93%	(36/39) 92.31%
*χ * ^2^-value	3.883	-	6.917	3.912
*P* value	0.002	-	0.001	0.002

## Data Availability

The data used to support the findings of this study are available from the corresponding author upon request.
